The article "Diagnostic Value of Color Doppler Flow Imaging Combined with Serum CRP, PCT, and IL-6 Levels for Neonatal Pneumonia" was retracted in 2023. Reasons: suspected computer-generated content; unreliable results or conclusions; concerns about the data; concerns about the results or conclusions.

# Diagnostic Value of Color Doppler Flow Imaging Combined with Serum CRP, PCT, and IL-6 Levels for Neonatal Pneumonia

**DOI:** 10.1155/2022/2113856

**Published:** 2022-08-10

**Authors:** Wenru Chen, Xiaoqing Yu

**Affiliations:** Fuzhou Children's Hospital of Fujian Medical University, Fuzhou 350004, China

## Abstract

**Objective:**

To evaluate the diagnostic value of combined detection of color Doppler flow imaging (CDFI) and serum C-reactive protein (CRP), procalcitonin (PCT), and interleukin-6 (IL-6) levels for neonatal pneumonia.

**Methods:**

In this prospective study, 30 newborns with pneumonia and 30 healthy newborns in our hospital from January 2019 to January 2020 were recruited. The healthy newborns were assigned to the control group, and the newborns with pneumonia were assigned to the experimental group. All subjects underwent CDFI and measurement of the levels of serum CRP, PCT, and IL-6. The serum indices and imaging results of the two groups were analyzed, and the specificity and sensitivity of different detection methods in the diagnosis of neonatal pneumonia were calculated and analyzed.

**Results:**

The levels of serum CRP, PCT, and IL-6 in the experimental group were significantly higher than those in the control group (*P* < 0.001). Combined detection had a larger detection area, higher sensitivity, and a superior overall detection outcome than single detection (*P* < 0.05). The diagnostic results of combined detection and clinical diagnosis in 30 newborns with pneumonia were similar (*P* > 0.05).

**Conclusion:**

The combined detection of CDFI and serum CRP, PCT, and IL-6 levels in the diagnosis of neonatal pneumonia shows a promising diagnostic outcome, so it is worthy of clinical application.

## 1. Introduction

Neonatal pneumonia is a common disease in neonatology, which refers to lung inflammation caused by bacteria in the newborn during or after delivery [1, 2]. Relevant studies have shown that neonatal pneumonia is an important factor for neonatal death, with a mortality rate between 5% and 20% [2–4]. The early onset of neonatal pneumonia is mostly accompanied by nonspecific symptoms. However, as the disease progresses, patients may experience symptoms such as cyanosis, dyspnea, and shortness of breath and become vulnerable to complications such as atelectasis and emphysema if timely and effective treatment is absent, which takes a toll on their life and health [5–7]. The current treatment mainly relies on comprehensive treatment methods to control inflammation, improve the lung ventilation function of patients, and mitigate clinical symptoms. Related studies have revealed that early diagnosis and treatment are of great significance to the prognosis of patients. With the continuous advancement of medical diagnostic technology, color Doppler flow imaging (CDFI) has been widely used in clinical diagnosis, providing a reference for following treatment [8, 9]. In addition, based on CDFI, the detection of serum C-reactive protein (CRP), procalcitonin (PCT), and interleukin-6 (IL-6) levels contributes to enhancing the diagnostic accuracy of neonatal pneumonia. Accordingly, the present study was conducted to further explore the diagnostic value of the combined detection of CDFI and serum CRP, PCT, and IL-6 levels for neonatal pneumonia.

## 2. Materials and Methods

### 2.1. General Information

In this prospective study, 30 newborns with pneumonia and 30 healthy newborns in our hospital from January 2019 to January 2020 were recruited. The healthy newborns were assigned to the control group, and the newborns with pneumonia were assigned to the experimental group.

### 2.2. Inclusion Criteria

Children who met the diagnostic criteria for neonatal pneumonia, who have not received imaging examinations and have not been treated, and whose parents provided written informed consent were included. This study was approved by the Fuzhou Children's Hospital, Fujian Medical University Ethics Committee (2019-2-417).

### 2.3. Exclusion Criteria

Children who were seriously ill and required a ventilator for treatment, with severe kidney, liver, and other organ dysfunction, and with immune system diseases were excluded.

## 3. Methods

All participants received CDFI (Beijing Kuntaide Medical Technology Co., Ltd.; C9). The examination was performed to obtain the lung images of the participants in three different positions, namely, sitting position, supine position, and prone position.

Inspection procedures: each chest wall of the participant was divided into three parts: anterior, lateral, and posterior part, and each part was divided into an upper part and a lower part. Overall, each chest wall was divided into 6 areas, with a total of 12 areas on both sides. All the intercostals in each area of the lungs were scanned to obtain the lesion status and determine the location, blood flow, and area of the lung consolidation. The existence of effusion in the chest cavity of the children was observed and recorded.

The early morning fasting cubital venous blood of all participants was collected, and the serum was centrifugated to collect the supernatant which was then stored at −80°C for the assay. The serum CRP, PCT, and IL-6 levels in the blood samples were determined according to the ELISA kit instructions. The specific steps are as follows: ① Sample dilution: the standards and the blood samples were diluted according to the instructions. ② Sample addition: blank holes, standard holes, and test holes were set without contaminating the ELISA plate. The standards of different concentrations were added to the standard wells, and 50 *μ*l/well of diluted serum was added to the test wells. The plate was then sealed with sealing tapes and incubated at 37°C for 60 minutes. ③ Plate rinsing: the concentrated washing liquid was diluted with double distilled water, followed by the removal of the sealing tape and the liquid in the wells. The prepared rinsing solution was added to each well and rested still for 1 min, followed by the removal of the rinsing solution by flicking the microtiter plate over a sink, and the remaining drops were dried by patting the plate on a paper towel. The operation was repeated 5 times. ④ Biotinylation working solution addition: 50 *μ*l of biotinylation working solution was added to each well, and the plate was sealed and incubated at 37°C for 30 minutes. Then, the same plate washing operation was conducted and repeated 5 times. The remaining drops were removed by patting the plate. ⑤ Enzyme conjugate working solution addition: 50 *μ*l of an enzyme conjugate was added to each well. Then, the plate was sealed and incubated at 37°C for 30 minutes. ⑥ Plate rinsing: the operation method and steps were the same as above and repeated 5 times. ⑦ Color development: 50 *μ*l of the color developer was added to each reaction well, shaken, mixed well, and placed in the dark at 37°C for 30 minutes for color development. ⑧ Reaction termination: 50 *μ*l of stop solution was added to each reaction well and mixed well to stop the reaction. ⑨ Microplate reader measurement: the absorbance value at 450 mm wavelength was measured within 15 minutes, and the absorbance value of each well was recorded.

All the above tests were completed in the laboratory of our hospital, and the detailed process is shown in Figure 1.

In addition, nebulized inhalation treatment of the 20 ml Huatan Pingchuan Decoction daily could be given (Ephedrae Herba, Earthworm, Pepperweed Seed, Asari Radix et Rhizoma, Belamcandae Rhizoma, Flos Farfarae, Almond, Semen Ginkgo, Stiff Silkworm, Safflower) with 7 days as one course.

### 3.1. Observational Indicators

The serum CRP, PCT, and IL-6 levels and combined diagnosis of the two groups of newborns were compared, and the specificity and sensitivity of different detection methods in the diagnosis of neonatal pneumonia were calculated.

CDFI diagnostic criteria: lung consolidation: a hypoechoic area sonogram appears, with similar echogenicity to liver echogenicity, the disappearance of gas strong echogenicity, and unclear boundary. Pleural effusion: internal segregation of pulmonary solids is present with no echo expectation and clear transmissions [10, 11]. The normal reference range of serum CRP: 0 mg/L–5 mg/L and >5 mg/L is considered positive. The normal reference range of PCT: 0 ng/L–5 ng/L and >5 ng/L is considered positive. The normal reference range of IL-6: 5 pg/mL–15 pg/mL and >15 pg/mL is considered positive.

### 3.2. Statistical Analysis

In this research, the data were analyzed using SPSS20.0 software, and GraphPad Prism 7 (GraphPad Software, San Diego, USA) was used to plot the graphics. The count data are expressed as [*n* (%)] and analyzed by the chi-square test, and measurement data are expressed as (mean ± SD) and analyzed by the *t*-test and normality test. The area under the curve (AUC) was calculated using the receiver operating curve (ROC). *P* < 0.05 indicated that the difference was statistically significant.

## 4. Results

### 4.1. Comparison of General Information

The two groups showed no significant differences in gender, average month age, BMI, Apgar score, and place of residence (*P* > 0.05) (Table 1).

### 4.2. Comparison of Serum Index Levels

The experimental group had significantly higher levels of serum CRP, PCT, and IL-6 than the control group (*P* < 0.05) (Figure 2).

### 4.3. Comparison of Single and Combined Detection of CDFI and Serum Indices

In comparison with single detection, combine detection had a larger detection area, as shown in Figure 3.

### 4.4. Comparison of the Area of Each Indicator, Standard Error^a^, Asymptotic Sig.^b^, and Asymptotic 95% Confidence Interval

Table 2 revealed better detection results in combined detection than single detection (*P* < 0.05).

### 4.5. Comparison of Sensitivity and 1-Specificity

The combined detection showed the highest sensitivity, as shown in Table 3.

### 4.6. Combined Detection Diagnosis of 30 Newborns with Pneumonia

There were no significant differences between the combined detection diagnosis and clinical diagnosis of 30 newborns with pneumonia (*P* > 0.05) (Table 4).

## 5. Discussion

Neonatal pneumonia refers to the inflammation of the lungs in children within 28 days of birth, and its cause is related to the underdevelopment of the respiratory function of the children [10, 12]. Ineffective treatment predisposes to disease recurrence, which hinders the growth and development of the children. In addition to anti-infective therapy, the regulation of inflammatory mediators is considered a new target for treating the disease [13–15]. Studies have found that early diagnosis has far-reaching significance for the prognosis of children. Serum CRP, PCT, and IL-6 indexes are common inflammatory factors and can directly reflect the inflammatory status of the body [16–18]. As a common clinical diagnostic method, CDFI is characterized by rapidness, noninvasiveness, easy operation, and high accuracy. It can obtain relevant information about the lesion by analyzing the ultrasound diagnosis data of the physiological and tissue structure. With regard to neonatal pneumonia, CDFI can accurately reflect the location and area of lung lesions and pleural effusion in the body, which provides an accurate basis for following treatment. The results of the present study showed that the serum CRP, PCT, and IL-6 levels of the experimental group were significantly higher than those of the control group (*P* < 0.05), which was consistent with the results of SLOOTWEG et al. [19] whose article demonstrated that “the levels of serum CRP, PCT, and IL-6 indexes in the observation group were (4.67 ± 2.02) mg/L, (0.49 ± 0.23) ug/L, and (23.04 ± 7.55) pg/mL, respectively, which were significantly higher than those of the control group (2.13 ± 0.41) mg/L, (0.08 ± 0.03) ug/L, and (8.51 ± 2.79) pg/mL, respectively (*P* < 0.05).” The results suggest that compared with healthy newborns, pneumonia is associated with inflammatory responses. Accordingly, serum CRP, PCT, and IL-6 indexes show great potential as important indicators for the diagnosis of neonatal pneumonia.

As a common inflammatory marker, the duration of an increased CRP level and its rate of elevation are related to the severity of inflammatory responses [20–22]. PCT is a sensitive indicator of bacterial infection. IL-6 is a lymphokine produced by activated T cells and fibroblasts, which promotes the differentiation of primitive bone marrow-derived cells and enhances the lysis function of natural killer cells [23]. However, the sensitivity of stand-alone detection of serum inflammatory factors or a single indicator level clinically was lower than that of the combined detection of CDFI and serum CRP, PCT, and IL-6 indexes. Furthermore, there were no significant differences between the combined detection diagnosis and clinical diagnosis of 30 children with pneumonia (*P* > 0.05). Taken together, combined detection shows a better detection outcome than single detection.

Apolipoprotein E (ApoE) gene polymorphisms in children's peripheral serum correlate with the presence of Mycoplasma pneumoniae infection in pediatric patients. The *ε*3 in the ApoE gene may have a protective effect against pediatric Mycoplasma pneumoniae infection, while *ε*4 may play a role in the pathogenesis of pediatric Mycoplasma pneumoniae infection, so research on these two aspects may provide a basis for targeted therapy.

## 6. Conclusion

In summary, combined detection of CDFI and serum CRP, PCT, and IL-6 levels shows high sensitivity and can provide a reliable reference basis for the later treatment of patients, which is worthy of promotion and application. Traditional Chinese medicine has made great progress in the treatment of neonatal pneumonia, with safe use and innovative routes of administration. However, the studies are mostly limited to clinical efficacy reports, lacking a strict scientific research design and an objective basis for experimental studies, resulting in inaccurate evaluation of efficacy. Therefore, further experimental studies on the treatment of this disease by traditional Chinese medicine should be conducted in the future to provide a scientific basis for clinical use.

## Figures and Tables

**Figure 1:** Research flow diagram.

**Figure 2:** Comparison of serum index test results between the two groups of research subjects. Note: the abscissa represents the diagnosis, and the ordinate represents the serum index; the serum CRP, PCT, and IL-6 levels of the experimental group after diagnosis were (6.88 ± 2.23) mg/L, (1.11 ± 0.28) ug/L, and (30.33 ± 8.24) pg/mL, respectively; serum CRP, PCT, and IL-6 levels of the control group after diagnosis were (2.15 ± 0.37) mg/L, (0.05 ± 0.02) ug/L, and (8.66 ± 2.68) pg/mL, respectively; the serum CRP levels of the two groups of subjects after diagnosis were significantly different (*t* = 14.062, ^*∗*^*P* < 0.05); the serum PCT levels of the two groups of subjects after diagnosis were significantly different (*t* = 20.683, ^*∗∗*^*P* < 0.01); the serum IL-6 levels of the two groups of subjects after diagnosis were significantly different (*t* = 13.698, ^*∗∗∗*^*P* < 0.001).

**Figure 3:** Comparison of single and combined detection of CDFI and serum indexes.

**Table 1:** Comparison of general information of the two groups of children [*n* (%)].

	Experimental group (*n* = 30)	Control group (*n* = 30)	*X* ^2^/*t*	*P*
Gender			0.067	0.795
Male	16 (56.25)	17 (56.67)		
Female	14 (43.75)	13 (43.33)		
Mean month age (d)			0.120	0.905
	11.27 ± 1.31	11.31 ± 1.27		
BMI (kg/m^2^)			0.069	0.945
	17.55 ± 3.42	17.49 ± 3.31		
Apgar scores			0.038	0.969
	6.51 ± 2.11	6.53 ± 1.98		
Place of residence			0.073	0.787
Urban	20 (56.25)	19 (50.00)		
Rural	10 (43.75)	11 (50.00)		

**Table 2:** Comparison of the area of each indicator, standard error a, asymptotic Sig.b, and asymptotic 95% confidence interval.

Variables of detection results	AUC	Standard error^a^	Asymptotic Sig.^b^	Asymptotic 95% confidence interval	
				Lower limit	Upper limit
CRP	0.727	0.068	0.003	0.594	0.860
PCT	0.709	0.069	0.006	0.574	0.845
IL-6	0.675	0.071	0.021	0.536	0.815
CDFI	0.711	0.069	0.005	0.576	0.846
CRP + PCT + IL-6	0.745	0.066	0.001	0.615	0.875
CDFI + CRP	0.744	0.066	0.001	0.614	0.874
CDFI + PCT	0.830	0.057	0.001	0.718	0.942
CDFI + IL-6	0.881	0.049	0.001	0.785	0.977
Combined detection	0.949	0.033	0.001	0.001	1.000

**Table 3:** Comparison of sensitivity and 1-specificity.

Variables of detection results	Positive^a^ if greater or equal to	Sensitivity	1-specificity
CRP	−1.0000 0.5000 2.0000	1.000 0.621 0.001	1.000 0.167 0.001

PCT	−1.0000 0.5000 2.0000	1.000 0.552 0.001	1.000 0.133 0.001

IL-6	−1.0000 0.5000 2.0000	1.000 0.517 0.001	1.000 0.167 0.001

CDFI	1.0000 0.5000 2.0000	1.000 0.655 0.001	1.000 0.233 0.001

CRP + PCT + IL-6	1.0000 0.5000 2.0000	1.000 0.690 0.001	1.000 0.200 0.001

CDFI + CRP	1.0000 0.5000 2.0000	1.000 0.621 0.001	1.000 0.133 0.001

CDFI + PCT	1.0000 0.5000 2.0000	1.000 0.793 0.001	1.000 0.133 0.001

CDFI + IL-6	1.0000 0.5000 2.0000	1.000 0.862 0.001	1.000 0.100 0.001

Combined detection	1.0000 0.5000 2.0000	1.000 0.966 0.001	1.000 0.067 0.001

**Table 4:** Combined detection diagnosis of 30 newborns with pneumonia.

Diagnosis method	*n*	Correctly diagnosed	Misdiagnosis, missed diagnosis	Correct diagnosis rate
Clinical diagnosis	30	100% (30/30)	0.00% (0/30)	100% (30/30)
Combined detection diagnosis	30	93.33% (28/30)	6.67% (2/30)	93.33% (28/30)
*x* ^2^				2.069
*P*				0.150

## Data Availability

All data generated or analysed during this study are included within this published article.
